The article "Effect of lncRNA PVT1/miR186/KLF5 Axis on the Occurrence and Progression of Cholangiocarcinoma" was retracted in 2024. Reasons: signs of a paper mill; compromised peer review; unreliable results or conclusions.

# Effect of lncRNA PVT1/miR186/KLF5 Axis on the Occurrence and Progression of Cholangiocarcinoma

**DOI:** 10.1155/2021/8893652

**Published:** 2021-07-10

**Authors:** Qiang Sun, Xueyi Gong, Jianlong Wu, Zhipeng Hu, Qiao Zhang, Jingling Gong, Xiaofeng Zhu

**Affiliations:** ^1^General Surgery Department, Zhongshan Hospital, Sun Yat-Sen University, Zhongshan, China; ^2^Organ Transplant Center, The First Affiliated Hospital of Sun Yat-Sen University, Guangzhou, China

## Abstract

This study primarily focused on the effect of the long noncoding RNA (lncRNA) PVT1/miR186/KLF5 axis on the occurrence and progression of cholangiocarcinoma (CCA). miR186 was found both in the lncRNA PVT1 targeting miRNAs and KLF5 targeting miRNAs using bioinformatic analysis. The expression of lncRNA PVT1 and KLF5 in the TFK-1, QBC939, and HuCCT1 cell lines and normal biliary epithelial HIBEpiC cells was detected by RT-qPCR. The significance of lncRNA PVT1 and KLF5 on cell proliferation was analyzed using the MTT assay and clone formation assay in lncRNA PVT1 and KLF5 silencing HuCCT1 cell lines and lncRNA PVT1and KLF5 overexpressing TFK-1 and QBC939 cell lines, respectively. The potential role of lncRNA PVT1 and KLF5 in cell migration was detected using the transwell invasion assay in CCA cell lines and tumor formation assay. Additionally, lncRNA PVT1 and KLF5 were proved to be highly expressed in CCA tissues and cell lines. Silencing and overexpressing of lncRNA PVT1 or KLF5 markedly inhibited or increased the cell proliferation and cell invasion in CCA cell lines, respectively. Silencing and overexpressing of lncRNA PVT1 significantly inhibited and increased the expression of KLF5 in CCA cell lines, respectively. Silencing of lncRNA PVT1 increased the expression of miR186, and silencing of miR186 increased the expression of KLF5 in CCA cell lines. Cotransfection of lncRNA PVT1 and miR186 increased the expression of KLF5 compared with controls. Overall, these results demonstrated that the lncRNA PVT1/miR186/KLF5 axis might exert a key role in the occurrence and progression of CCA, and this axis might provide a new target for treating CCA.

## 1. Introduction

Cholangiocarcinoma (CCA) is a common epithelial cancer with a very poor survival rate and a poor overall prognosis because of limited treatment options [1, 2]. CCA can be divided into intrahepatic, perihilar, and distal CCA which refer to the anatomical location [3]. The incidence of CCA in Asian countries is clearly higher than that in other areas; however, it has become more and more common in Europe and North America [4]. Surgical treatment is the most primary option for all types of CCA, but it is still difficult to cure CCA because of the majority of the patients diagnosed with CCA in the advanced stage [5]. Based on the abovementioned background, it is necessary to clarify the potential molecular mechanisms in CCA pathogenesis and search for new biomarkers that may serve as potential therapeutic targets of CCA.

The article "Effect of lncRNA PVT1/miR186/KLF5 Axis on the Occurrence and Progression of Cholangiocarcinoma" was retracted in 2024. Reasons: signs of a paper mill; compromised peer review; unreliable results or conclusions.

Long noncoding RNAs (lncRNAs) belong to the noncoding RNA (ncRNA) family with length exceeding 200 nt. Although lacking protein-coding potential, lncRNAs play an essential role in cell proliferation, development, and differentiation by serving as significant regulators in the gene expression networks [6, 7]. Recently, the roles of lncRNAs in the occurrence and development of multiple cancer types have been substantiated, including colorectal cancer, breast cancer, ovarian cancer, prostate cancer, CCA, and melanoma [8]. The lncRNA PVT1 oncogene is located at 8q24.21, the downstream of *MYC* gene, and has been reported overexpressed in multiple cancer types and acts as a credible predictor of poor prognosis and overall survival rate [9–11]. Recently, Yu's group discovered that the expression of lncRNA PVT1 was dramatically enhanced in CCA, and the biological functions of lncRNA PVT1 in CCA have been demonstrated [12]. The transcription factor KLF5 in the WNT signaling pathway was reported upregulated in the CCA progression and growth [13]. Tang's group demonstrated that lncRNA PVT1 promoted proliferation and tumorigenesis in triple-negative breast cancer (TNBC) by the PVT1–KLF5-*β*–catenin axis, providing the first direct evidence of the association between lncRNA PVT1 and KLF5 in breast cancer [14]. According to the above facts, we hypothesized that the association between lncRNA PVT1 and KLF5 was essential in the occurrence and progression of CCA. Using bioinformatic analysis, we discovered that miR186 was found in both lncRNA PVT1 and KLF5 signaling pathways. Therefore, the lncRNA PVT1/miR186/KLF5 axis may be a novel signaling pathway that participates in CCA progression.

Herein, we primarily focused on the expression of lncRNA PVT1 and KLF5 in CCA and elucidated the effect of the lncRNA PVT1/miR186/KLF5 axis on the occurrence and progression of CCA and provided valuable insights into the therapeutic strategy of CCA.

## 2. Materials and Methods

### 2.1. Sample Acquisition and Cell Culture

In this work, CCA tissue samples and adjacent normal tissues were collected from 25 patients who were undergoing clinical surgery, and informed consent was obtained in Zhongshan Hospital (Zhongshan, China). The collected tissue samples were immediately frozen and maintained at -80°C after excision to extract RNA and perform RT-qPCR. The present work was approved by the Ethics Committee of Sun Yat-Sen University. CCA cell lines TFK-1, QBC939, and HuCCT1 and normal biliary epithelial HIBEpiC cells were grown in RPMI-1640 medium (Hyclone, Cat.No.SH30809.01B) containing 10% FBS (Hyclone, Cat.No.SH30087.01) and were cultivated at 37°C in a humidified 95% air and 5% CO_2_.

The article "Effect of lncRNA PVT1/miR186/KLF5 Axis on the Occurrence and Progression of Cholangiocarcinoma" was retracted in 2024. Reasons: signs of a paper mill; compromised peer review; unreliable results or conclusions.

### 2.2. Quantitative Real-Time Polymerase Chain Reaction (qRT-PCR)

A Takara reverse transcription kit was used to synthesize the first strand of cDNA. The kit was used to perform the real-time PCR process with the following reaction conditions: 95°C for 2 min, then a three-step PCR program for 40 cycles (95°C for 15 sec, 62°C for 32 sec). The specificity of the amplified products was determined by the melting curve analysis. The data were collected and analyzed by the ABI PRISM® 7500 Sequence Detection System. The relative expression of mRNA was obtained according to the Ct value automatically analyzed by the system. The following are the lncRNA sequences: PVT1 primer sequences, forward 5′-TTGCTGCTAGTGGACATGAG-3′ and reverse 5′-CAGTAGCCTCAGTGAACTCC-3′; KLF5 primer sequences, forward 5′-AGCAGCAATGGACACTCTTA-3′ and reverse 5′-GAAACTGACTTGGCATTGTG-3′; and miR186 primer sequences, forward 5′-ACACTCCAGCTGGGCAAAGAATTCTCCTTTTG-3′ and reverse 5′-CTCAACTGGTGTCGTGGA-3′.

### 2.3. Plasmid Construction and Cell Transfection

To construct the lncRNA PVT1, miR186, and KLF5 silenced cell lines, small interfering RNA (siRNA) was synthesized by XX company targeting the above genes. The siRNA sequences were as follows: lncRNA PVT1, sense, 5′ GUGUUAUUUGAGUCCAUCAdTdT-3′, antisense, 5′ UGAUGGACUCAAAUAACACdTdT-3′; miR186, sense, 5′-3′, antisense, 5′-3′; and KLF5, sense, 5′-3′, antisense 5′-3′. Scramble (NC) primer sequences are forward, 5′ UUCUCCGAACGUGUCACGUTT-3′, reverse, 5′ ACGUGACACGUUCGGAGAATT-3. To construct the lncRNA PVT1 and KLF5 overexpressed cell lines, sequences coding lncRNA PVT1 and KLF5 were subcloned to pCDH lentivectors.

For cell transfection, the siRNAs were transfected to CCA cell lines using Lipofectamine RNAi MAX (Thermo Fisher Scientific). pCDH lentivectors were transfected into CCA cell lines with pMD2.G and psPAX2 using Lipofectamine 2000 (Invitrogen, Cat.No. 11668019).

### 2.4. MTT Experiment

Briefly, 1 × 10^4^ cells/well were placed in 96-well plates after 24 h of cell transfection. 24 h after incubation, the supernatant was discarded and cells were dispersed in 100 *μ*l RPMI-1640 which contains 10% FBS. 10 *μ*l CellTiter96AQ (Promega, Cat.No.G3582) was added and incubated for 4 h. After 4 h incubation, the absorbance of cells was observed at 490 nm by the Multiskan MK3 plate reader (Thermo Fisher Scientific) for the cell proliferation rate evaluation.

The article "Effect of lncRNA PVT1/miR186/KLF5 Axis on the Occurrence and Progression of Cholangiocarcinoma" was retracted in 2024. Reasons: signs of a paper mill; compromised peer review; unreliable results or conclusions.

### 2.5. Colony Formation Experiment

CCA cell lines from different transfected groups were inoculated into a 6-well plate at 1 × 10^3^/well and incubated for about 2 weeks to observe colony formation. The cells were placed in 4% PFA for staining with a crystal violet reagent. The number of cell clones could be observed and calculated via microscope imaging.

### 2.6. Transwell Experiment

The upper chamber was inoculated with CCA cell lines (1 × 10^5^) from different transfected groups that were suspended in 100 *μ*l serum-free RPMI-1640 medium. The lower chamber was filled with 600 *μ*l RPMI-1640 medium supplemented with 10% FBS and incubated 24 h, and then, the cells were removed which are on the upper surface of the insert. The cells on the bottom surface were immobilized in 4% PFA for staining with crystal violet, and the cell number of migration cells was counted under a microscope.

### 2.7. Tumor Formation Experiment

All experimental procedures were compliant with the Sun-Yet Sen University and in accordance with the National Institutes of Health *Guide for the Care and Use of Laboratory Animals*. All mice were housed under specific pathogen-free conditions with an alternating 12 h light/dark cycle at 25 ± 2°C and provided with free access to autoclaved food and water. After acclimatization for at least 1 week, mice were randomly divided into 6 groups (three mice per group): HuCCT1 cells of NC group, siKLF5 group; TKF1 cells of NC group and KLF5OE group; and QBC939 cells of NC group and KLF5OE group. Then, each mouse was inoculated with 1 × 10^6^ transfected cells by subcutaneous injection into the dorsal flanks of nude mice. The tumor size was measured every 2 days from the third day after injection by the use of a digital caliper, and the tumor volume was determined with the following formula: tumor volume (mm^3^) = (length (mm)) × (width [mm])^2^ × 0.52. Thirty-five days after tumor cell implantation, all mice were sacrificed by CO_2_ inhalation to ameliorate animal suffering, and tumor xenografts were excised and weighed.

### 2.8. Dual-Luciferase Reporter Assay

lncRNA PVT1 fragments or KLF5 fragments with 3′ UTR were subcloned to luciferase plasmid psiCHECKTM-2 (Promega, C8011). The miR186 was subcloned to pCDH lentivectors. XX was used as a control luciferase plasmid. The recombinant plasmids were cotransfected into CCA cell lines that were incubated in 24-well plates. After 24 h transfection, the cells were harvested and lysed with Passive Lysis Buffer. After centrifugation, the supernatants were collected and the luciferase activity was determined under a dual-luciferase assay reporter system (GloMax™ 20/20, Promega) following the manufacturer's manual.

The article "Effect of lncRNA PVT1/miR186/KLF5 Axis on the Occurrence and Progression of Cholangiocarcinoma" was retracted in 2024. Reasons: signs of a paper mill; compromised peer review; unreliable results or conclusions.

### 2.9. Western Blotting

The cells were gathered and lysed with the standard lysis buffer after 48 h transfection. After centrifugation, the supernatants were collected for the measurement of protein concentration. The expression levels of KLF5 in different CCA cell lines were measured by Western blot as mentioned above. The primary antibodies were anti-KLF5 (Abcam, ab24331) and anti-GAPDH (Kangcheng, KC-5G5). Images were acquired by ChemiDoc MP (Bio-Rad).

### 2.10. Statistical Analysis

Using GraphPad Prism 8.0 software, the data was analyzed which is expressed as the mean ± standard deviation. The paired data significance was calculated using an independent samples *t*-test. All experiments were repeated 3 times. *p* > 0.05 was indicated statistically significant.

## 3. Results

### 3.1. lncRNA PVT1 Is Upregulated in CCA Tissues and Cell Lines

In order to explore the role of lncRNA PVT1 in CCA, we detected the expression level of lncRNA PVT1 in CCA tissues and adjacent normal tissues from 25 patients with CCA via RT-qPCR. Additionally, the expression levels of lncRNA PVT1 in 3 CCA cell lines and normal biliary epithelial HIBEpiC cells were analyzed. The results revealed that the expression level of lncRNA PVT1 was dramatically higher in CCA cell lines compared with the control group. Meanwhile, the patients with higher lncRNA PVT1 expression exhibited poorer survival rates. The data indicated that the progression of CCA was associated with upregulated lncRNA PVT1 expression (Figure 1).

### 3.2. Positive Regulation of lncRNA PVT1 on Cell Proliferation

To identify the functional role of lncRNA PVT1 on cell proliferation, the clone formation assay and MTT assay were conducted to evaluate the cell proliferation rate in CCA cell lines. The silencing effect of lncRNA PVT1 on the HuCCT1 cell line and the overexpression of lncRNA PVT1 in TFK-1 and QBC939 cell lines were quantified by RT-qPCR (Figure 2(a)). The data indicated that the cell proliferation rate and clone formation ability were markedly lower in the lncRNA PVT1 silencing group in the HuCCT1 cell line; however, it was remarkably higher in the lncRNA PVT1 overexpressing group in TFK-1 and QBC939 cell lines (Figures 2(b)–2(d)). The statistical data analysis of the data revealed that lncRNA PVT1 positively regulated the cell proliferation of CCA cell lines.

### 3.3. Positive Regulation of lncRNA PVT1 on Cell Migration

To investigate the role of lncRNA PVT1 in cell migration, the transwell invasion assay was used to detect the cell invasion behavior of CCA cell lines. It was found that the number of cells in the lncRNA PVT1 silencing group in the HuCCT1 cell line passing through Matrigel was remarkably lower than that in the NC group, whereas it was remarkably higher in the lncRNA PVT1 overexpressing group in TFK-1 and QBC939 cell lines (Figures 3(a) and 3(b)).

The article "Effect of lncRNA PVT1/miR186/KLF5 Axis on the Occurrence and Progression of Cholangiocarcinoma" was retracted in 2024. Reasons: signs of a paper mill; compromised peer review; unreliable results or conclusions.

### 3.4. Positive Regulation of lncRNA PVT1 on the Growth of Xenografts in Nude Mice

To further investigate the vital role of lncRNA PVT1 in vivo, we injected the lncRNA PVT1 silenced and overexpressed CCA cell lines into nude mice and then observed the growth of xenografts. As illustrated in Figures 3(c) and 3(d), the average volume and weight of the tumors in the lncRNA PVT1 silenced group were markedly decreased; however, they were significantly increased in the lncRNA PVT1 overexpressed groups. Thus, these results clearly showed that lncRNA PVT1 positively regulated CCA tumor growth in vivo.

### 3.5. Expression of KLF5 in CCA Tissues and Cell Lines

In order to explore the vital role of KLF5 in CCA, the expression level of KLF5 in CCA tissues and adjacent normal skin tissues from 25 patients with CCA was detected via RT-qPCR. To evaluate the relationship between lncRNA PVT1 and KLF5, the expression level of KLF5 was detected in lncRNA PVT1 silenced and overexpressed CCA cell lines. In Figure 4(a), the expression level of KLF5 in CCA tissues was dramatically higher than that in normal tissues (control group). The expression level of KLF5 was dramatically lower in the lncRNA PVT1 silenced group; however, it was significantly higher in lncRNA PVT1 overexpressed groups (Figure 4(b)). Collectively, these obtained data indicated showed that the progression of CCA was related to the upregulated KLF5, and lncRNA PVT1 positively regulated the expression of KLF5 in CCA cell lines.

### 3.6. Positive Regulation of KLF5 on Cell Proliferation

To identify the essential role of KLF5 in cell proliferation, the cell proliferation rate in CCA cell lines was analyzed using the MTT assay and clone formation assay. Our data indicated that the cell proliferation rate and clone formation ability were clearly lower in the KLF5 silenced group. They were significantly higher in the KLF5 overexpressed groups compared to control groups (Figures 5(a)–5(d)). Therefore, these findings further confirmed that KLF5 positively regulated cell proliferation of CCA cell lines.

### 3.7. Effects of lncRNA PVT1/miR186/KLF5 Axis on CCA Cell Lines

To identify the relationship of the lncRNA PVT1/miR186/KLF5 axis, the direct interaction between lncRNA PVT1 and miR186 and between miR186 and KLF5 was detected by a dual-luciferase reporter assay (Figure 6(a)). Additionally, we analyzed the expression level of miR186 in lncRNA PVT1 silenced CCA cell lines and the expression of KLF5 in miR186 silenced groups using RT-qPCR. Moreover, we determined the expression of KLF5 in CCA cell lines cotransfecting with lncRNA PVT1 and miR186 using Western blot analysis. It was found that the expression level of miR186 in lncRNA PVT1 silenced groups was apparently higher compared to NC groups (Figure 6(b)). The expression of KLF5 in miR186 silenced groups was dramatically higher compared to NC groups (Figure 6(c)). Cotransfection of lncRNA PVT1 and miR186 increased the expression of KLF5 compared with controls (Figure 6(d)). Taken together, these results indicated that the lncRNA PVT1/miR186/KLF5 axis might contribute to the occurrence and development of CCA.

The article "Effect of lncRNA PVT1/miR186/KLF5 Axis on the Occurrence and Progression of Cholangiocarcinoma" was retracted in 2024. Reasons: signs of a paper mill; compromised peer review; unreliable results or conclusions.

### 3.8. Positive Regulation of KLF5 on Cell Migration and the Growth of Xenografts in Nude Mice

In Figures 7(a) and 7(b), the number of cells in the HuCCT1 cell line passing through Matrigel was apparently decreased in the KLF5 silenced group compared with the NC group; however, it was significantly higher in the KLF5 overexpressed group in TFK-1 and QBC939 cell lines. In addition, the average volume and weight of the tumors in the KLF5 silenced group were dramatically enhanced, but they were markedly increased in the KLF5 overexpressed groups (Figures 7(c) and 7(d)). These results indicated that KLF5 positively regulated cell migration and tumor growth in CCA.

## 4. Discussion

This study primarily focused on the essential role of the lncRNA PVT1/miR186/KLF5 axis in the development and progression of CCA. In this work, it was shown that the expression of lncRNA PVT1 and KLF5 in the CCA tissues and cell lines was remarkably increased as compared to the adjacent normal tissues and control cells. Silenced lncRNA PVT1 and KLF5 apparently inhibited cell proliferation, migration, and the growth of xenografts in nude mice. However, the overexpressed lncRNA PVT1 and KLF5 significantly increased cell proliferation, cell migration, and the growth of xenografts in nude mice. Meanwhile, miR186 was found in both lncRNA PVT1 and KLF5 signaling pathways. The interactions between lncRNA PVT1 and miR186, and miR186 and KLF5, were confirmed using a dual-luciferase reporter assay. Furthermore, silenced lncRNA PVT1 remarkably increased the expression of miR186, and silenced miR186 significantly increased the expression of KLF5; cotransfection of lncRNA PVT1 and miR186 increased the expression of KLF5 compared with controls. Collectively, these results indicated that the lncRNA PVT1/miR186/KLF5 axis may take an essential role in the occurrence and progression of CCA.

lncRNA PVT1 is an essential noncoding RNA that lies in well-known cancer risk locus [15] and has been proved involved in different cancer types, including breast and ovarian cancers [16], acute myeloid leukemia [17], prostate cancer [18], and thyroid carcinoma [19]. The essential role of lncRNA PVT1 in CCA progression and inflammation was demonstrated through a genome-wide lncRNA screening [20]. And the biological functional role of lncRNA PVT1 in CCA has been demonstrated recently, but the underlying mechanism of the effects of overexpression has not been determined [12]. This study indicated that lncRNA PVT1 was significantly increased in the CCA tissues and cell lines compared with the control group, indicating that the role of lncRNA PVT1 in CCA cell proliferation and migration has been demonstrated.

The article "Effect of lncRNA PVT1/miR186/KLF5 Axis on the Occurrence and Progression of Cholangiocarcinoma" was retracted in 2024. Reasons: signs of a paper mill; compromised peer review; unreliable results or conclusions.

KLF5 belongs to the zinc-finger-containing transcription factor family participating in gene regulation and was found overexpressed in various human cancers, affecting several signaling pathways associated with cancer [21]. For instance, KLF5 promotes thyroid cancer tumorigenesis and metastatic potential through the NF-*κ*B signaling pathway [22]. KLF5 could potentially contribute to cell proliferation, and cell invasion of cervical cancer partly relies on TNFRSF11a expression [23]. In addition, KLF5 promotes cell proliferation and cell invasion of breast cancer partially dependent on the transcription of TNFAIP2 [24]. KLF5 in the WNT signaling pathway was reported upregulated in the CCA progression and growth [13]. Collectively, these data indicated that KLF5 was overexpressed in the CCA tissues and cell lines, and the key role of KLF5 in CCA cell proliferation and migration has been demonstrated.

Tang's group discovered that lncRNA PVT1 could contribute to proliferation and tumorigenesis in TNBC dependent on the PVT1–KLF5-*β*–catenin axis, demonstrating the association between lncRNA PVT1 and KLF5 in breast cancer [14]. Since lncRNA PVT1 and KLF5 were significantly overexpressed in CCA tissues and cell lines, we thereby hypothesized that these two molecules belong to the same pathway affecting the occurrence and development of CCA. We used the bioinformatic analysis to predict the possible lncRNA PVT1 targeting miRNAs and the miRNAs that might be aimed at regulating KLF5 function, and we discovered that one of the miRNAs, namely, miR186, was found in both clues, indicating the potential role of the lncRNA PVT1/miR186/KLF5 axis in the progression of CCA.

To further explore the roles of lncRNA PVT1 and KLF5 in CCA, silenced and overexpressed CCA cell lines were constructed to evaluate their effects on CCA cell proliferation, cell migration, and tumorigenesis. The results revealed that silenced lncRNA PVT1 and KLF5 obviously inhibited cell proliferation, clone formation, cell migration, and the growth of xenografts in nude mice. However, the overexpressed lncRNA PVT1 and KLF5 have significantly opposite effects. Collectively, these results clearly indicated that abnormal expression of lncRNA PVT1 and KLF5 plays a vital role in promoting cell proliferation, cell migration, and tumorigenesis of CCA.

The article "Effect of lncRNA PVT1/miR186/KLF5 Axis on the Occurrence and Progression of Cholangiocarcinoma" was retracted in 2024. Reasons: signs of a paper mill; compromised peer review; unreliable results or conclusions.

To confirm the lncRNA PVT1/miR186/KLF5 axis in this study, the interaction between lncRNA PVT1 and miR186 was determined through a dual-luciferase reporter assay, miR186 and KLF5. The obtained data indicated that lncRNA PVT1 interacted with miR186, and miR186 interacted with KLF5, providing powerful evidence for the identification of the lncRNA PVT1/miR186/KLF5 axis. The role of lncRNA PVT1 in regulating miR186 expression was further demonstrated using lncRNA PVT1 silenced CCA cell lines. The findings suggest that silenced lncRNA PVT1 substantially increased the expression of miR186. In addition, the role of miR186 in regulating KLF5 expression was confirmed using miR186 silenced CCA cell lines. The results showed that silenced miR186 clearly promoted the expression of KLF5. Moreover, the cotransfection of lncRNA PVT1 and miR186 increased the expression of KLF5 compared with controls. Overall, these results demonstrated the essential role of the lncRNA PVT1/miR186/KLF5 axis in the occurrence and progression of CCA.

In conclusion, both in vitro and in vivo studies documented the essential role of lncRNA PVT1 and KLF5 in the occurrence and progression of CCA. Moreover, the role of the lncRNA PVT1/miR186/KLF5 axis was confirmed in CCA cell lines, which may be a novel signaling pathway that contributes to CCA development.

## Figures and Tables

**Figure 1:** Expression of lncRNA PVT1 in CCA: (a) lncRNA PVT1 expression in CCA tissues and (b) cell lines quantified by qRT-PCR. ^∗^*p* < 0.05.

**Figure 2:** Effects of lncRNA PVT1 on cell proliferation of CCA. (a) The silencing effect of lncRNA PVT1 on HuCCT1 cells and the overexpression of lncRNA PVT1 in TFK-1 and QBC939 cells were quantified by RT-qPCR. (b) Cell proliferation activity by MTT assay of cells in different groups. (c, d) The cell colony activity of different cells. siPVT1: silenced PVT1 cells; OE: overexpression. ^∗^*p* < 0.05.

**Figure 3:** Effects of lncRNA PVT1 on cell migration of CCA. (a, b) Role of PVT1 in cell migration in HuCCT1, TFK-1, and QBC939 cells. (c, d) The growth of xenografts in nude mice 30 days after transplantation. OE: overexpression. ^∗^*p* < 0.05.

**Figure 4:** Expression of KLF5 in CCA. (a) KLF5 expression in CCA tissues. (b) The expression of KLF5 in lncRNA PVT silenced HuCCT1 cell and lncRNA PVT overexpressed TFK-1 and QBC939 cells were quantified by Western blot. OE: overexpression. ^∗^*p* < 0.05.

The article "Effect of lncRNA PVT1/miR186/KLF5 Axis on the Occurrence and Progression of Cholangiocarcinoma" was retracted in 2024. Reasons: signs of a paper mill; compromised peer review; unreliable results or conclusions.

**Figure 5:** Effects of KLF5 on cell proliferation of CCA. (a) The silencing effect of KLF5 on HuCCT1 cells and the overexpression of KLF5 in TFK-1 and QBC939 cells were quantified by Western blot. (b) Silenced KLF5 significantly inhibited HuCCT1 cell proliferation, and overexpressed KLF5 significantly increased TFK-1 and QBC939 cell proliferation measured by MTT experiment. (c, d) Silenced KLF5 markedly decreased the number of HuCCT1 cell colonies, and overexpressed KLF5 significantly increased the number of TFK-1 and QBC939 cell colonies. OE: overexpression. ^∗^*p* < 0.05.

**Figure 6:** Identification of lncRNA PVT1/miR186/KLF5 axis. (a) Quantification analysis of interaction between lncRNA PVT1 and miR186 measured by dual luciferase assay. (b) Silenced lncRNA PVT1 markedly increased the expression of miR186. (c) Silenced miR186 clearly increased the expression of KLF5. (d) The expression of KLF5 after cotransfection of lncRNA PVT1 and miR186 (OE). ^∗^*p* < 0.05.

**Figure 7:** Effects of KLF5 on cell migration of CCA. (a, b) Silenced KLF5 significantly decreased the number of HuCCT1 cell migration, and overexpressed KLF5 significantly increased the number of TFK-1 and QBC939 cell migration. (c, d) The growth of xenografts in nude mice 30 days after transplantation. OE: overexpression. ^∗^*p* < 0.05.

## Data Availability

All data, models, and code generated or used during the study appear in the submitted article.
